# Analysis of Different Vascular Accesses on Dialysis Quality and Infection Risk Factors of Hemodialysis Patients

**DOI:** 10.1155/2021/4554417

**Published:** 2021-08-26

**Authors:** Huaping Wu, Xiang Li, Cunliang Zeng, Li Zhang, Huanhuan Song, Kaiping Lv

**Affiliations:** Department of Cardiac & Vascular Surgery, Dazhou Central Hospital, Dazhou, Sichuan 635000, China

## Abstract

**Objective:**

To explore the influence of different vascular accesses on dialysis quality and infection risk factors of hemodialysis patients.

**Methods:**

A total of 162 patients with end-stage renal disease admitted to our hospital from February 2018 to July 2020 were divided into two groups: cuff tunnel conduit (CTC) group and native arteriovenous fistula (AVF) group. Peripheral blood was collected before and 6 months after dialysis. The incidence of vascular recirculation was measured, and the risk factors of infection were analyzed.

**Results:**

The levels of HB, Alb, CRP, BUN, Scr, and TP after dialysis in the two groups were lower than those before dialysis (*P* < 0.05). The Kt/V of patients in both groups did not exceed 1.2, and the URR value exceeded 60%. The results of independent-samples *T* test analysis documented that the Kt/V level of patients in the AVF group was higher than that of those in the CTC group after dialysis (*P* < 0.05). The results of the urea method revealed that 22 of 68 patients (32.35%) in the CVC group and 21 of 94 (22.34%) in the AVF group had vascular pathway recirculation. The *χ*^2^ test showed that there was no remarkable difference in the incidence of vascular pathway recirculation between both groups (*P* > 0.05). However, the results of the nonurea method revealed that the incidence of vascular pathway recirculation in the AVF group was lower than that in the CVC group (*P* < 0.05). Multivariate logistic regression was used to further analyze the factors with statistical significance in the single factor results. It showed that age >60 years, dialysis duration >1 year, dialysis times, diabetes, hypertension, and CTC were all independent risk factors causing vascular access infection.

**Conclusion:**

If all conditions permit, AVF hemodialysis is a better choice for patients with end-stage renal disease. For the elderly, long-term hemodialysis, and those with diabetes and hypertension, it is necessary to make detailed plans, strengthen the operation proficiency of CTC, and reduce the incidence of infection.

## 1. Introduction

Hemodialysis is a vital treatment for all uremic patients to survive. For those who need dialysis for a long time, establishing and maintaining permanent vascular accesses with good function is a crucial condition for prolonging their survival [1, 2]. A stable and reliable vascular access is the basic guarantee for smooth hemodialysis. To achieve this goal, and to improve the dialysis effect and quality of life of patients, it is necessary to establish scientific vascular accesses according to patients' condition [3, 4].

Cuff tunnel conduit (CTC) and native arteriovenous fistula (AVF) are two kinds of vascular accesses frequently used in clinical practice, which have their own advantages and disadvantages [5, 6]. The advantage of CTC is that it is easy to operate and can be inserted into multiple catheters. CTC can improve the dialysis quality of hemodialysis patients and has less influence on hemodynamics. But the disadvantage is that it is easy to puncture the artery by mistake and cause hematoma. If the operation is not standardized and the disinfection is not in place, it is very easy to cause catheter-related infection, which leads to vascular endothelial damage and stenosis and then leads to thrombosis in the tube, which makes CTC lose its original function and even affects patients' extubation [7–9]. AVF is another method to establish vascular accesses rapidly. Related studies show that AVF is the best permanent vascular access in clinical application. Compared with CTC, AVF has the advantages such as long service life, stable blood flow, and low incidence of internal fistula infection and thrombosis [10, 11]. Once embolism occurs, it becomes extremely difficult to reconstruct internal fistula [12].

Therefore, it is increasingly important to choose which vascular access and how to maintain it in clinical treatment. At present, there are few comparative studies on the two. In addition, infection is the main cause of morbidity and death in patients with chronic hemodialysis [13]. It is also of great significance to confirm the risk factors of infection in patients with chronic long-term hemodialysis. On the basis of analyzing the therapeutic effects of these two kinds of vascular access, this study further analyzed the risk factors of vascular access infection in order to provide reference for clinical hemodialysis.

## 2. Materials and Methods

### 2.1. General Data

A total of 162 patients with end-stage renal disease admitted to our hospital from February 2018 to July 2020 were divided into CTC group (*n* = 68) and AVF group (*n* = 94) according to the vascular accesses established during hemodialysis. Inclusion criteria: all patients were over 18 years old and had been treated with maintenance hemodialysis for more than one month, and no dialyzer or pipeline coagulation occurred during dialysis treatment. Exclusion criteria: patients with hypotension, heart failure, painful spasm, etc., during dialysis treatment; those with systemic inflammatory reaction; those with liver cirrhosis; and pregnant or lactating women were excluded. This study has been approved by the Medical Ethics Committee of our hospital, and all patients have signed an informed consent form.

### 2.2. Therapeutic Methods

Patients in both groups were treated with the B Braun hemodialysis machine (Melsungen, Germany) and Fresenius F6 dialyzer (Bad Homburg, Germany). The dialysis frequency was 4 h three times a week, the blood flow rate was 250 mL/min, the dialyzate flow rate was 500 mL/min, and the dialyzate was bicarbonate dialyzate (Quinton, Virginia, USA) with a concentration of 34 mmol/L (potassium 2.0 mmol/L, calcium 1.5 mmol/L, and magnesium 0.5 mmol/L). Establishment of vascular accesses: patients in both groups were placed in a supine position, and after the arteriovenous vascular access was confirmed, lidocaine was used for local anesthesia; those in the CTC group were established with cuff tunnel catheter, model 13.6 F *∗* 36 cm (Joka Kathetertechnik, Hechingen, Germany); and those in the AVF group were established with autologous arteriovenous fistula. Anticoagulant method: the whole body heparinization method was used for anticoagulation. That is to say, heparin was used for the first time at 0.3–0.5 mg/kg and then maintained at 0.3–5 mg/kg during dialysis. The vascular access was established in the upper limbs of patients.

### 2.3. Evaluation of Dialysis Adequacy by Urea Clearance Index and Decline Rate

Peripheral blood was collected before and 6 months after dialysis. Hemoglobin (Hb), plasma albumin (Alb), total protein (TP), C-reactive protein (CRP), urea nitrogen (BUN), and creatinine (Scr) were detected using an automated blood and biochemical analyzer (Beckman Coulter, Beijing, China). The urea clearance index (Kt/V) and urea decline rate (URR) were calculated. Kt/V = −Ln(*R* − 0.008*t*) + (4 − 3.5*R*) *∗* UF/*W*, where *R* = urea nitrogen after permeation/urea nitrogen before permeation, *t* is the dialysis time (h), UF = ultrafiltration volume = volume before permeation − volume after permeation (L), and *W* is the body weight after permeation (kg). URR = 100/(1 − urea after permeation/urea before permeation).

### 2.4. Access Recirculation

The urea method was used to measure the incidence of vascular pathway recirculation. After dialysis for 30 min, ultrafiltration was stopped and blood was collected from the arterial end and venous end; blood flow was reduced to 100 mL·min^−1^ immediately after blood collection, blood pump was turned off after 10 s, arterial blood was collected from the contralateral artery, and dialysis was resumed. The recirculation rate was *R* = (Cs − Ca)/(Cs − Cv) × 100%, where Ca, Cv, and Cs are the concentrations of BUN in the artery, vein, and whole body serum, respectively. In the nonurea method, glucose injection was used to measure the pathway recirculation. After dialysis was performed for 30 min, the rotation speed of blood pump was 300 mL·min^−1^, ultrafiltration was closed, 0.1 mL arterial blood was collected, and blood glucose was measured using a blood glucose meter, which was *G*1 (mg·dL^−1^). Altogether 2 mL of 50% glucose injection and 3 mL normal saline were injected intravenously within 4 s, and 0.1 mL arterial blood was collected again within 13–17 s. The blood glucose *G*2 was measured. If *G*2 > *G*1, the recirculation rate (Ret) was calculated using the formula Ret = 0.046 (*G*2 − *G*1) + 0.07.

### 2.5. Infection Detection

According to the “Consensus of Experts on Vascular Access for Hemodialysis in China,” the blood samples of arterial and venous cavities and peripheral blood of patients suspected of vascular access infection were immediately collected for culture, and the pathogen results were identified. If the growth time of bacteria in catheters is earlier than that in peripheral blood for more than 2 h, it can be suspected of catheter-related infection. Patients with infection should be treated with empirical antibiotic before blood culture results are obtained, and then antibiotics should be selected according to blood culture and drug sensitivity test results. For local redness, blood clots, abscesses, etc., local ointment rubbing or incision drainage and continuous negative pressure suction should be adopted according to their severity. In addition, for those who fail in anti-infection treatment or whose access cannot be continued, total resection of artificial blood vessel, subtotal resection of artificial blood vessel, and partial resection of artificial blood vessel are used.

### 2.6. Statistical Analysis

SPSS19.0 was used for statistical analysis. The data conforming to normal distribution were expressed as mean ± standard deviation (SD), and the counting data were expressed as percentage. The statistical differences of counting data between the two groups were compared by the *χ*^2^ test, the differences of measurement data were compared by the *T* test, and the risk factors of vascular access infection were analyzed by logistic regression. *P* < 0.05 is considered a statistical difference.

## 3. Results

### 3.1. Analysis of Clinical Pathological Data of Patients

First, we compared the clinicopathological data of the two groups, including gender, age, dialysis duration and times, etc. After *χ*^2^ and independent-samples *T* tests, there was no statistical difference in the basic data between the two groups (all *P* > 0.05) (Table 1).

### 3.2. Changes of Biochemical Indexes before and after Dialysis in Both Groups

There was no obvious difference in HB, Alb, CRP, BUN, Scr, and TP between both groups before and after dialysis (*P* > 0.05), but their levels after dialysis were lower than those before (*P* < 0.05) (Table 2).

### 3.3. Evaluation of Dialysis Adequacy

We use Kt/V and URR to evaluate dialysis adequacy of the two groups of patients. In this research, the Kt/V of the two groups of patients did not exceed 1.2, and the URR value exceeded 60%. Independent-samples *T* test analysis documented that the Kt/V level of patients in the AVF group was higher than that of those in the CTC group after dialysis (*P* < 0.05), and there was no marked difference in URR (*P* > 0.05) (Figure 1).

### 3.4. Analysis of Vascular Pathway Recirculation in Two Groups of Patients

Recirculation of vascular access is a crucial reason that affects dialysis effect. Excessive recirculation will lead to the decline of dialysis efficiency. In this research, the detection results of vascular access recirculation by urea showed that 22 of 68 patients (32.35%) in the CVC group and 21 of 94 (22.34%) in the AVF group had vascular access recirculation. *χ*^2^ test results showed that there was no marked difference in the incidence of vascular pathway recirculation between the two groups (*P* > 0.05). However, the results of the nonurea method revealed that the incidence of vascular pathway recirculation in the AVF group was lower than that in the CVC group (*P* < 0.05) (Table 3).

### 3.5. Univariate Analysis of Vascular Access Infection

In this research, 31 patients had vascular access infection, and the incidence rate was 19.14%. Univariate analysis showed that the proportion of patients with diabetes, hypertension, acute cortical necrosis, and receiving CTC in the infected group was higher than that in the uninfected group (*P* < 0.05), and the dialysis frequency of the infected group was higher than that in the uninfected group (*P* < 0.05) (Table 4).

### 3.6. Multivariate Logistic Analysis of Vascular Access Infection

Multivariate logistic regression was used to further analyze the factors with statistical significance in the single factor results. It manifested that age >60 years, dialysis duration >1 year, dialysis times, diabetes, hypertension, and CTC were all independent risk factors causing vascular access infection (Table 5).

## 4. Discussion

Recently, with the increased incidence of chronic kidney disease, the number of patients with renal failure is gradually increasing [13]. To treat uremia caused by renal failure, hemodialysis is used more and more widely, and the advantages and disadvantages of various vascular pathways are more exposed to the vision of medical workers [5, 14]. To carry out hemodialysis smoothly, it is particularly important for long-term dialysis patients to make individualized dialysis plans reasonably and establish and maintain good functional vascular accesses [15].

At the moment, there are many kinds of vascular access used clinically, among which CTC and AVF are the most commonly used. CTC is especially used for patients who need hemodialysis urgently or in the short term but have no vascular access, but it also requires highly skilled medical workers. Irregular operation can easily cause catheter-related infection and catheter thrombosis, resulting in catheter failure [16, 17]. AVF has the advantages of stable blood flow, infection of internal fistula, and low incidence of embolism, but it cannot be used in emergency hemodialysis and can only be used after the internal fistula matures [10, 18]. Thus, these two methods are also used as complementary schemes to each other in clinical practice. In 2019, the National Kidney Foundation recommended AVF as the first choice of vascular access for children undergoing maintenance hemodialysis (HD) [19], but there are few data compared with other types of access. The results of this research showed that HB, Alb, CRP, BUN, Scr, and TP in CTC and AVF groups were improved after dialysis, but there was no statistical difference between both groups. After calculating Kt/V and URR, the Kt/V value of the AVF group was higher than that of the CTC group, which showed that AVF had better dialysis adequacy. Adequacy of dialysis is a vital index to evaluate the effective elimination of metabolites and the correction of electrolyte disorder by hemodialysis. Krzanowski et al. [20] found that the type of vascular pathway affected the infection complications and survival of hemodialysis patients. Compared with AVF, the infection rate and mortality of CTC patients are higher, and the prognosis of AVF patients is better. Hence, they think that AVF should be used in all possible situations. Jeong et al. [21] explained that there was a similar conclusion that the mortality of patients in the AVF group was lower than that of those in the CTC group, and they also confirmed that the first use of CVC was an independent risk factor leading to the decrease of the survival rate of patients.

Because of the short time of this research, we did not analyze the death of patients but analyzed the infection of vascular access. Infection is the main cause of morbidity and death of chronic hemodialysis patients, and the requirement of frequent catheter replacement also increases the cost of dialysis. In hemodialysis, the incidence of CTC infection increases with the extension of use time [22]. In our results, the incidence of infection in the AVF group was lower than that in the CTC group. Furthermore, age >60 years, dialysis duration >1 year, dialysis frequency, diabetes, hypertension, and CTC were independent risk factors for vascular access infection. Schwanke et al. [23] discovered that age and diabetes were the risk factors of central venous catheter infection in hemodialysis, so special attention should be paid to such patients to avoid infection. Therefore, our research is partially consistent with the above published experimental results.

Nevertheless, there are still some shortcomings mainly because the distribution of infected flora is not analyzed, and the nutritional status and personal hygiene of patients are not evaluated. In a prospective study, it is considered that maintaining good personal hygiene may be one of the most important measures to prevent infection of hemodialysis patients [24]. These shortcomings need to be further supplemented in our future research.

To sum up, if all conditions permit, it is a better choice to use AVF to treat patients with end-stage renal disease. For the elderly, long-term hemodialysis, and those complicated with diabetes and hypertension, it is necessary to make a detailed plan, strengthen the operation proficiency of CTC, and reduce the incidence of infection.

## Figures and Tables

**Figure 1:** Evaluation of dialysis adequacy of two groups of patients. (a) comparison of Kt/V between two groups. (b) comparison of URR value between two groups. ^*∗*^*P* < 0.05.

**Table 1:** Analysis of clinicopathological data of two groups of patients (*n*, $\bar{x}$ ± *s*, %).

	CTC group (*n* = 68)	AVF group (*n* = 94)	*χ*^2^/*t*	*P*
Gender			1.223	0.269
Man	46 (67.65)	71 (75.53)		
Woman	22 (32.35)	23 (74.47)		

Age			1.689	0.194
≤60 years old	35 (51.47)	58 (61.70)		
>60 years old	33 (48.53)	36 (38.30)		

Dialysis duration			0.861	0.353
≤1 year	28 (41.18)	32 (34.04)		
>1 year	40 (58.82)	62 (65.96)		

Dialysis times	24 ± 15	27 ± 12	1.413	0.160

Complicated with diabetes			1.220	0.269
Yes	13 (19.12)	12 (12.77)		
No	55 (80.88)	82 (87.23)		

Complicated with hypertension			0.256	0.613
Yes	16 (23.53)	19 (20.21)		
No	52 (76.47)	75 (79.79)		

Access location			0.809	0.369
Left arm	41 (60.29)	50 (53.19)		
Right arm	27 (39.71)	44 (46.81)		

Type of nephropathy			2.126	0.713
Chronic glomerulonephritis	48 (70.59)	71 (75.53)		
Diabetic nephropathy	8 (11.76)	10 (10.64)		
Chronic interstitial nephritis	6 (8.82)	7 (7.45)		
Hypertensive nephropathy	5 (7.35)	3 (3.19)		
Acute cortical necrosis	1 (1.47)	3 (3.19)		

Karnofsky score	82 ± 18	81 ± 20	0.327	0.744

**Table 2:** Changes of biochemical indexes before and after dialysis in both groups (*n*, $\bar{x}$ ± *s*).

		CTC group (*n* = 68)	AVF group (*n* = 94)	*t*	*P*
Hb (g/L)	Before dialysis	95.13 ± 9.53	96.56 ± 9.13	0.966	0.336
	After dialysis	93.25 ± 8.66^*∗*^	93.32 ± 9.37^*∗*^	0.048	0.961

Alb (g/L)	Before dialysis	45.21 ± 4.17	44.26 ± 5.11	1.256	0.210
	After dialysis	43.52 ± 4.58^*∗*^	42.43 ± 4.24^*∗*^	1.561	0.121

CRP (mg/L)	Before dialysis	17.35 ± 7.16	17.29 ± 6.83	0.054	0.957
	After dialysis	15.48 ± 7.13^*∗*^	16.05 ± 7.02^*∗*^	0.507	0.613

BUN (mmol/L)	Before dialysis	32.35 ± 8.16	32.52 ± 8.13	0.122	0.903
	After dialysis	8.15 ± 2.06^*∗*^	7.82 ± 2.05^*∗*^	1.009	0.315

Scr (*μ*mol/L)	Before dialysis	846.26 ± 207.53	854.13 ± 214.12	0.234	0.815
	After dialysis	226.15 ± 66.11^*∗*^	225.95 ± 70.58^*∗*^	0.018	0.985

TP (g/L)	Before dialysis	78.47 ± 6.33	79.34 ± 6.74	0.812	0.407
	After dialysis	76.54 ± 7.12^*∗*^	77.82 ± 6.41^*∗*^	1.197	0.233

*Note.*^*∗*^*P* < 0.05 after dialysis compared with before dialysis.

**Table 3:** Analysis of vascular pathway recirculation in two groups of patients (*n*, $\bar{x}$ ± *s*, %).

		CTC group (*n* = 68)	AVF group (*n* = 94)	2/*t*	*P*
Urea method	Happened	22	21	2.029	0.154
	Not happened	46	73		
	R	32.35%	22.34%		

Nonurea method	G1 (mg/dL)	113.76 ± 31.54	116.23 ± 21.37		
	G2 (mg/dL)	142.35 ± 51.17	124.71 ± 23.66		
	Ret (%)	1.414 ± 1.037	0.455 ± 0.124	8.889	<0.001

**Table 4:** Univariate analysis of vascular access infection (*n*, $\bar{x}$ ± *s*, %).

	Infection (*n* = 31)	No infection (*n* = 131)	*χ* ^2^	*P*
Gender			1.135	0.287
Man	20 (64.52)	97 (74.05)		
Woman	11 (35.48)	34 (25.95)		

Age			12.624	<0.001
≤60 years old	9 (29.03)	84 (64.12)		
>60 years old	22 (70.97)	47 (35.88)		

Dialysis duration			5.140	0.023
≤1 year	6 (19.35)	54 (41.22)		
>1 year	25 (80.65)	77 (58.78)		

Dialysis times	30 ± 18	21 ± 13	3.696	<0.001

Complicated with diabetes			90.598	<0.001
Yes	22 (70.97)	3 (2.29)		
No	9 (29.03)	128 (97.71)		

Complicated with hypertension			72.809	<0.001
Yes	20 (64.52)	15 (11.45)		
No	11 (35.48)	116 (88.55)		

Access location			0.324	0.569
Left arm	16 (51.61)	75 (57.25)		
Right arm	15 (48.39)	56 (42.75)		

Type of nephropathy			17.778	0.001
Chronic glomerulonephritis	20 (64.52)	99 (75.57)	1.572	0.210
Diabetic nephropathy	4 (12.90)	14 (10.69)	0.125	0.724
Chronic interstitial nephritis	2 (6.45)	11 (8.40)	0.139	0.720
Hypertensive nephropathy	1 (3.23)	7 (5.34)	0.239	0.625
Acute cortical necrosis	4 (12.90)	0 (0.00)	Fisher	0.001
Karnofsky score	77 ± 12	85 ± 17	3.326	0.001

Vascular access mode			41.864	<0.001
CTC	29 (93.55)	39 (29.77)		
AVF	2 (6.45)	92 (70.23)		

**Table 5:** Multivariate logistic analysis of vascular access infection.

Variable		Wald	OR	95%CI	*P*
Age (years)	>60 vs. ≤60	4.793	2.246	1.583–2.437	0.038
Duration of dialysis (years)	>1 vs. ≤1	5.246	2.718	2.385–3.461	0.032
Dialysis times		4.317	2.234	1.383–2.847	0.042
Diabetes	Yes vs. No	18.074	8.327	8.185–9.333	0.012
Hypertension	Yes vs. No	9.274	4.291	4.315–5.368	0.015
Type of nephropathy	Acute cortical necrosis vs. others	8.045	3.268	3.214–3.893	0.056
Karnofsky score		12.315	5.783	3.156–5.743	0.057
Vascular access mode	CTC vs. AVF	4.356	2.383	1.736–2.748	0.023

## Data Availability

The data used are available from the corresponding author.
